# Application of Deep Learning Technology in Glioma

**DOI:** 10.1155/2022/8507773

**Published:** 2022-02-18

**Authors:** Guangdong Hu, Fengyuan Qian, Longgui Sha, Zilong Wei

**Affiliations:** Department of Neurosurgery, Shanghai Pudong Hospital, Fudan University Pudong Medical Center, Pudong, Shanghai 201399, China

## Abstract

A common and most basic brain tumor is glioma that is exceptionally dangerous to health of various patients. A glioma segmentation, which is primarily magnetic resonance imaging (MRI) oriented, is considered as one of common tools developed for doctors. These doctors use this system to examine, analyse, and diagnose appearance of the glioma's outward for both patients, i.e., indoor and outdoor. In the literature, a widely utilized approach for the segmentation of glioma is the deep learning-oriented method. To cope with this issue, a segmentation of glioma approach, i.e., primarily on the convolution neural networks, is developed in this manuscript. A DM-DA-enabled cascading approach for the segmentation of glioma, which is 2DResUnet-enabled model, is reported to resolve the problem of spatial data acquisition of insufficient 3D specifically in the 2D full CNN along with the core issue of memory consumption of 3D full CNN. For gliomas segmentation at various stages, we have utilized multiscale fusion approach, attention, segmentation, and DenseBlock. Moreover, for reducing three dimensionalities of the Unet model, a sampling of fixed region is used along with multisequence data of the glioma image. Finally, the CNN model has the ability of producing a better segmentation of tumor preferably with minimum possible memory. The proposed model has used BraTS18 and BraTS17 benchmark data sets for fivefold cross-validation (local) and online evaluation preferably official, respectively. Evaluation results have verified that edema's Dice Score preferable average, enhancement, and core areas of the segmentation of the glioma with DM-DA-Unet perform exceptionally well on the validation set of BraTS17. Finally, average sensitivity was observed to be high as well, which is approximately closer to the best segmentation model and its effect on the validation set of BraTS1 and has segmented gliomas accurately.

## 1. Introduction

For providing facilities for doctors to remove gliomas of brain precisely and accurately during the surgery, images play a vital role in the clinical treatment, i.e., computed tomography (CT), positron emission computed tomography (PET), and magnetic resonance imaging (MRI). Learn imaging technology to segment the brain glioma area, so as to help doctors to remove brain tumors efficiently and accurately in the largest range [1–5].

Likewise, MRI possesses contrast of soft tissue and has the ability of providing information about rich physiological tissues. Therefore, for treatment of glioma, MRI is utilized for the preoperative diagnosis, intraoperative treatment, and postoperative review of glioma. As glioma is defined as a tumor which consists of multiple tumor tissues (such as necrotic core, tumor active edge, and edema tissue), multiple sequences of MRI are utilized to image various brain tumor tissues.

The segmentation of glioma and its surrounding tissues (particularly abnormal), i.e., MRI-enabled, is more feasible for doctors in the observation process of external morphology where every tumor tissue of patients with glioma appears, and it is also helpful for doctors to conduct image-oriented analysis and further analysis of gliomas. Hence, glioma segmentation is assumed as the very basic step in the analysis of MRI which is related to the glioma patients. Gliomas have various malignant degrees and multiple tumor tissue areas. At the same time, brain MRI is a multimodal three-dimensional scan image with a large number of layers, so manual segmentation of the glioma area requires a lot of time and manpower. Additionally, traditional segmentation, i.e., manual, is primarily based on image's brightness which is observed through the eyes of human, and image generation is a common factor to affect its quality. Additionally, annotator's personal factors result in quality of segmentation which is uneven, incorrect, and redundant. Thus, a completely automatic approach of segmentation specifically with exceptional accuracy of glioma is desperately required to carry out segmentation of glioma in the clinical practice. Glioma segmentation approach, which is based on the deep learning, may resolve the issues of manual analysis of data and design segmentation features in traditional image processing algorithms and machine learning algorithms and can automatically segment gliomas, which greatly overcomes the brain. The shortcomings of glioma segmentation that require strong prior constraints and manual intervention improve the robustness and effectiveness of the algorithm and can achieve better segmentation results in large-scale multimodal and complex glioma segmentation scenes [6–10].

The rest of the manuscript is arranged according to the following agenda items.

A brief literature review is presented along with various issues associated with the existing state-of-the-art approaches described. In Section 3, the proposed deep learning enabled diagnosis method is described in detail sufficiently where every term is described. Experimental results and observations are presented where comparative study is depicted to describe usefulness of the proposed scheme against state-of-the-art existing approaches. Lastly, concluding remarks are provided at the end.

## 2. Related Work

During the last two or three decades, a subbranch of the artificial intelligence, i.e., deep learning, has become an integral approach to resolve numerous complex operations or tasks with high accuracy. Among these approaches, CNN which is proposed by LeCun and Bengio has made great progress in the field of image processing [11]. Therefore, segmentation methods based on convolutional neural networks are widely used in medical image segmentation tasks and have achieved good segmentation results in lung nodule, retinal, liver cancer, and brain segmentations of glioma [12].

In the segmentation method of glioma based on convolutional nerve, a traditional method is to use CNN to classify each pixel in the patient's MRI so as to distinguish the glioma area and the background area and achieve the purpose of glioma segmentation. The neural network used in this segmentation method is called a convolutional neural network for pixel-by-pixel segmentation. Among the convolutional neural networks for pixel-by-pixel segmentation, Zikic et al. first used convolutional neural networks to solve the problem of brain glioma segmentation [13], using a 5-layer 2D CNN structure to segment multimodal glioma images. Devorak and Menze proposed a CNN segmentation method based on small image blocks [14], which made the model pay more attention to the local structural features of glioma. Havaei et al. proposed a brain cancer segmentation method based on a dual-path convolutional neural network [15], with two two-dimensional input images of different sizes. The input image with a larger size is used as the input of the first path convolutional neural network, and another feature map with the same size is obtained after the model prediction is output. Then, merge the two feature maps as the input of the second path CNN and finally output the segmentation result of the pixel. At the same time, Pereira et al. trained two CNN [16], which were used to segment high-grade gliomas and low-grade gliomas. And use morphological methods to postprocess the segmentation results to remove false positive pixels in the segmentation results.

Different from the general full CNN, Ronneberger et al. proposed a symmetric full CNN called Unet [17]. It has achieved convincing performance on medical images and has been widely used in various tasks. On the basis of the original Unet structure, Dong et al. proposed a 2DUnet structure based on two-dimensional convolution [18] and used it in automatic brain tumor segmentation. In order to increase the spatial information acquisition capability of the Unet structure, Beers et al. replaced the two-dimensional convolution in Unet with three-dimensional convolution [19]. A fully convolutional network called 3DUnet is proposed and used in glioma segmentation. However, due to the small number of layers of the original Unet structure and small image input, the 2DUnet and 3Dunet proposed on the original Unet structure both have weak feature extraction capabilities and poor segmentation effects for high-resolution images.

In addition to brain glioma segmentation, related researchers have proposed many improved structures based on Unet and used them in image segmentation tasks in various fields. The Res-Unet [20] network was inspired by ResNet [21], replacing each submodule in the original Unet structure with residual connection blocks and achieved a good segmentation effect in the segmentation task of retinal blood vessels. Dense-Unet [22] is used to remove artifacts in medical images. This model is inspired by DenseNet [23], replacing each submodule in the original Unet with densely connected blocks, thereby improving the segmentation effect. Attention Unet [24] introduced an Attention mechanism in Unet. Before splicing the corresponding features of each stage in the downsampling encoding part and the upsampling decoding part, an attention module was used to readjust the encoding in the upsampling process. This structure is used in the segmentation task of CT abdominal images.

## 3. Segmentation Method of Glioma Based on DM-DA-Unet

Considering that the two-dimensional fully convolutional network has the characteristics of low memory consumption, fast prediction speed, and high sensitivity, the three-dimensional fully convolutional network is sensitive to spatial information and can effectively train and predict three-dimensional data. This chapter proposes a DM-DA-Unet (Dual Multidimensional Dense Attention Unet) network structure for glioma segmentation in a cascaded manner. This structure uses full convolutional networks of different dimensions to segment brain gliomas at different stages, which can effectively improve the segmentation accuracy of brain gliomas.

### 3.1. Network Structure

Since the brain MRI in the BraTS data set is a thin-slice MRI, the layer thickness on the *z*-axis is only 1mm, and the number of layers in the image is 155, so the brain MRI in the BraTS data set has rich spatial information. However, two-dimensional convolution can only perform feature extraction on each layer of a three-dimensional image, so it is easy to lose the spatial information of the glioma, which reduces the segmentation effect of the glioma. The three-dimensional convolution can convolve the input three-dimensional data in three directions (*x*, *y*, and *z*) to extract features. Therefore, the neural network using three-dimensional convolution can obtain more than the neural network using two-dimensional convolution. Spatial features are better for segmentation of three-dimensional data.

However, in brain glioma segmentation, the input brain MRI data has a large three-dimensional size. If you directly use three-dimensional convolution to extract features from the entire brain MRI data, the input size and output size of the model will be too large. Therefore, a large amount of computer video memory is consumed in the process of model training and prediction, resulting in the general hardware environment being unable to conduct model training and testing at all. At the same time, the use of larger-sized three-dimensional data as model input will also cause serious imbalance between positive and negative samples, slow training time, difficulty in model debugging, and huge amount of model parameters. In response to the above problems, on the basis of 2DResUnet, this paper proposes the use of different dimensional convolutions for feature extraction at different stages. The DM-DA-Unet structure for segmentation of glioma regions in a cascade manner is shown in Figure 1.

In the two stages of the network cascade mechanism, a full convolutional network of different dimensions is used to segment the glioma. In the first stage, 2DDenseUnet is used to locate the glioma area. In the second stage, the 3D-DA-Unet structure was used to accurately segment the glioma. Among them, the DenseBlock mechanism is used in both 2DDenseUnet and 3D-DA-Unet.

This is because the residual mechanism of ResNet will merge the output of the previous layer *H*_*i*_(*X*_*i*−1_) and the identity map *X*_*i*−1_ directly through addition, which will limit the flow of the gradient. Therefore, in order to improve the flow of gradients between different layers in the network, DenseNet [23] uses a different connection method. The output before the *i*-th layer is connected to the *i*-th layer through identity mapping, thereby making the connection between layers in the network closer. In this connection mechanism, the *i*-th layer in DenseNet can be expressed as

(1) $$\begin{array}{c} X_{i}=H_{i}\left(\left[X_{0},X_{1},\ldots ,X_{i-1}\right]\right), \end{array}$$

where [•] represents the layer-to-layer concatenation, which is to concatenate the feature maps output from the 0th layer to the *i* − 1 th layer in the network.

The connection mechanism of the above DenseNet is generally called DenseBlock. DenseBlock can solve the problem of gradient disappearance more effectively than ResBlock while increasing the depth of the network and can enhance the reuse and propagation of features. Therefore, replace the ResBlock block in 2DResUnet with the DenseBlock block to design the 2DDenseUnet model. And, on the basis of 2DDenseUnet, the three-dimensional convolution and Attention mechanism are applied to the Unet structure to design a 3D-DA-Unet model. And because the original DenseNet is designed for the classification task of natural images, it contains several maximum pooling layers, which may cause the loss of shallow feature information in the high-resolution feature map. Therefore, in the two subnetworks of DM-DA-Unet, a convolutional layer with a step size of 2 is used to downsample the image, thereby reducing the loss of shallow features.

### 3.2. 2DDenseUnet Structure

In 2DDenseUnet, the Encoder DenseBlock structure is shown in Figure 2. The structure consists of three convolution kernels with a size of 3*∗*3 and a two-dimensional convolution with a step size of 1, as well as a BN layer and PReLU activation function. And through the concatenation mechanism to connect the front and back layer features, this connection method allows the input features of the last convolutional layer in Encoder DenseBock to be spliced by the feature maps output by all the convolutional layers.

The Decoder DenseBlock structure mainly includes a two-dimensional convolutional layer with a size of 3*∗*3 and a step size of 1 by three convolution kernels. A convolution kernel used to extract features of the input is a 1 × 1 two-dimensional convolution with fixed bias. The concatenation mechanism is used to make dense connections between the various layers, as shown in Figure 3.

### 3.3. 3D-DA-Unet Structure

In DM-DA-Unet, 3D-DA-Unet is used to accurately segment gliomas using three-dimensional convolution in the second stage. The 3D-DA-Unet network consists of the downsampling part of the encoded image, the upsampling part of the decoded image, the multiscale fusion mechanism, and the Attention mechanism of the features before and after the connection. Among them, the downsampling part includes 1 3D Input Module structure, 3 3D DenseBlock structures, and 3 three-dimensional convolutions with a step size of 2. Among them, the three-dimensional convolution with a step size of 2 is used to downsample the feature map. The upsampling part consists of 3 3D upsampling layers, 3 3D Localization Module structures, and 1 3D Output Module structure. The 3D upsampling layer is used for the upsampling of feature maps. The Attention mechanism consists of a main branch and a Soft Mask Branch, which are used to fuse the features of the downsampling part and the upsampling part of the model. The multiscale fusion part collects feature maps of different scales at various stages during the upsampling process and scales their sizes to the same scale through upscale and adds them to the final output feature map to fuse multiscale features. In 3D-DA-Unet, when the image passes through the three-dimensional convolutional layer, the Instance Nomalization layer is often used for feature normalization, and the Leaky ReLU activation function is used to add nonlinear features.

Since the traditional BN layer calculates the mean and variance through batch size data, it is more sensitive to the batch size of the image input. In glioma segmentation, because the glioma image is a multisequence image, if the batch size is too large, it will cause memory leaks and insufficient video memory. Therefore, a smaller batch size is generally used for training and prediction, and the batch size is too large. Small will cause the mean and variance calculated by the BN layer not to conform to the distribution of the original image. Therefore, in 3D-DA-Unet, the IN layer is needed to standardize the input image instances, which can not only accelerate the model convergence, but also maintain the independence in each image instance.

At the same time, because the commonly used activation function ReLU sets all the negative values in the feature map to zero, for standardized glioma input, there are intensity values less than 0. Therefore, it is necessary to use Leaky ReLU to assign a nonzero slope to all negative variables, so as to eliminate the disappearance of the gradient caused by the use of the ReLU function. In the 3D-DA-Unet network structure, the 3D Input Module is used to extract features of the input image and add it to the network backbone. It consists of an image input layer, a three-dimensional convolution with a convolution kernel size of 3*∗*3*∗*3 and a step size of 1, an IN layer for feature map normalization, and an activation function Leaky ReLU.

The 3D DenseBlock structure is a coding structure that extracts image features during the 3D-DA-Unet downsampling process, which includes two sets of three-dimensional convolution, IN layer and the feature extraction structure composed of the activation function Leaky ReLU, and uses the concatenation mechanism to stitch the structure, before and after the features, thereby constructing the DenseBlock structure.

The 3D Localization Module structure is that 3D-DA-Unet merges the feature map obtained by the Attention mechanism and the feature map amplified by the 3D upsampling layer during the upsampling process. And the number of channels is reduced by the three-dimensional convolution with the size of the convolution kernel of 1*∗*1*∗*1, thereby reducing the amount of parameters in the training process. At the same time, in order to increase the depth of the structure, a simple residual block is constructed through the ADD mechanism.

The 3D Output Module is composed of a multiscale fusion feature map, the size of the convolution kernel is 1*∗*1*∗*1, the number of convolution kernels is the number of glioma regions, a three-dimensional convolution with a step size of 1, and a Sigmoid activation function. This structure is used to fuse the feature maps of various scales generated during the feature upsampling process and finally output the prediction results of the model; that is, the feature maps after the Sigmoid activation function are the probability maps of the model prediction results.

### 3.4. Attention Mechanism

In the traditional Unet structure, the connection between the downsampling encoding part and the upsampling decoding part is often through the concatenation mechanism to directly splice the front and back features, so there is a problem of insufficient feature extraction of the downsampling part in the splicing process.

This article uses ResBlock-based Attention mechanism in 3D-DA-Unet to connect the downsampling part and upsampling part of the network structure. At the same time, considering the increase in the amount of parameters brought by the Attention mechanism and the problem of large memory consumption, the complexity of the Attention mechanism is simplified. Therefore, the Attention mechanism used in 3D-DA-Unet is shown in Figure 4. The Attention mechanism includes a main branch and a Soft Mask Branch. Among them, the main branch is used to learn original features, and the Soft Mask Branch is used to reduce noise and enhance features.

In the Attention mechanism of 3D-DA-Unet, the feature map of each size generated in the downsampling process will first be extracted through a three-dimensional convolution with a convolution kernel size of 3*∗*3*∗*3. Then, input the extracted features into the two branches of the Attention mechanism, namely, into the Trunk Branch and the Soft Mask Branch at the same time.

In Trunk Branch, the original input features are extracted through a ResBlock structure using three-dimensional convolution. The ResBlock structure consists of two three-dimensional convolution kernels with a size of 3*∗*3*∗*3 and a step size of 1, the corresponding IN layer, and the Leaky ReLU layer. It can effectively perform deep feature extraction on the original features and output the extracted feature maps.

The Soft Mask Branch uses the same features as the Trunk Branch, through a three-dimensional convolution with a convolution kernel size of 3*∗*3*∗*3 and a step size of 1 as well as a convolution kernel with a size of 1*∗*1*∗*1 and a step size of 1 to obtain the feature map. And use the Sigmoid activation function to control the intensity value of the feature map before 0 to 1, so as to obtain a feature map for suppressing the output noise of Trunk Branch.

After obtaining the output feature maps of Trunk Branch and Soft Mask Branch, first multiply the output feature maps of Trunk Branch and Soft Mask Branch through a multiplication operation. Then, add the result of the multiplication and the output of the Trunk Branch to get the feature map of the Attention mechanism, as shown in the formula:

(2) $$\begin{array}{c} OA=\left(1+S\left(x\right)\right)T\left(x\right), \end{array}$$

where *OA* represents the output of the Attention mechanism, *x* represents the input feature map, *S*(*x*) represents the output feature map of Soft Mask Branch, and *T*(*x*) represents the output feature map of Trunk Branch. This superposition method can effectively suppress the noise in the output feature map of Trunk Branch and extract the original features to the greatest extent, which can enhance the depth of the network while reducing information loss.

The feature information extracted by the Attention mechanism will be fused with the feature map of the corresponding size in the upsampling, so as to ensure the effective feature connection between the downsampling part and upsampling part.

### 3.5. Loss Function

For DM-DA-Unet, since it uses two-dimensional convolutional network models in two stages, in the training process of the model, it is necessary to use different loss functions to train the two network models. For 2DDenseUnet, the loss function used is the sum of GDL (Generalised Dice Loss) and WCE (Weighted Cross Entropy) as the loss function.

The calculation method of GDL is shown in the following formula:

(3) $$\begin{array}{c} \mathrm{GDL}=1-2\frac{\sum_{l=1}^{L}w_{l}\sum_{n}^{N}r_{\ln}p_{\ln}}{\sum_{l=1}^{L}w_{l}\sum_{n}^{N}r_{\ln}+p_{\ln}}, \end{array}$$

where *L* represents the number of label categories, *N* represents the number of pixels, *p*_*ln*_ represents the pixel value of the prediction result, *r*_*ln*_ represents the pixel value of the real mask, and *w*_*l*_ represents the weight of each category, which can be expressed as

(4) $$\begin{array}{c} w_{l}=\frac{1}{{\left(\sum_{l=1}^{N}r_{\ln}\right)}^{2}},\\ \mathrm{WCE}=-\frac{1}{N}\sum_{n=1}^{N}\sum_{l=1}^{L}\left[w_{l}r_{n}\log\;p_{n}+\left(1-r_{n}\right)\log\left(1-p_{n}\right)\right], \end{array}$$

where *L* represents the label category, *N* represents the number of pixels, *r* represents the mask label, *p* represents the model segmentation result, and *w* represents the weight of the label.

For 3D-DA-Unet, due to the unevenness of the three-dimensional samples in the three-dimensional glioma data and the difficulties caused by multiregion segmentation, therefore, Weighted Dice Loss (WDL) is used as the loss function in the training process. The formula is as follows:

(5) $$\begin{array}{c} \mathrm{GDL}=-\frac{1}{4}\sum_{l=1}^{L}\frac{\left(2\sum_{n}^{N}\left(r_{\ln}p_{\ln}+\mathrm{smooth}/2\right)\right)}{\sum_{n\mathrm{=1}}^{N}r_{\ln}+\sum_{n\mathrm{=1}}^{N}p_{\ln}+\mathrm{smooth}}, \end{array}$$

where *L* is the number of categories, *N* is the number of pixels, *r* is the real mask label, *p* is the model prediction result, and smooth is the smoothing factor. Because the loss function not only considers the intersection ratio of the three-dimensional segmentation mask and the real mask, but also combines the segmentation results of the four segmented regions at the same time, therefore, the loss function can alleviate the imbalance of positive and negative categories in the three-dimensional data, and consider the division of multiple regions at the same time.

### 3.6. Segmentation Algorithm

The overall process of the glioma segmentation method based on DM-DA-Unet can be described as follows:

1. The first step is to separately preprocess the data input to the two subnetworks of DM-DA-Unet. For the 3D-DA-Unet model, based on the idea of cascading segmentation, a method of using fixed region sampling in the model training and prediction process is proposed to obtain the three-dimensional cube data for 3D-DA-Unet training.
2. The second step is to perform data enhancement on the preprocessed image. In the 3D-DA-Unet model, in order to make full use of the spatial information in the three-dimensional input data, the data enhancement method of TTA (Test Time Augmentation) is used. The three-dimensional rotation is used to enhance the data during training and prediction, thereby significantly improving the segmentation accuracy of 3D-DA-Unet.
3. The third step is to perform model training. Since the model is a cascade model, two of the models need to be trained separately. For 2DDenseUnet, each layer in the training data needs to be trained during the model training process. Sampling is performed to complete the sampling of the overall input data. 3D-DA-Unet only needs to use the three-dimensional cube data with the glioma center as the sampling center and the sampling size of 128*∗*128*∗*128 for training and prediction, so as to accurately segment the glioma in a fixed area.
4. The fourth step is to evaluate the performance of the trained model. The evaluation indicators used are Dice Score, sensitivity, specificity, and Hausdorff distance.
5. The fifth step is the process of predicting data, which is different from the end-to-end model structure such as 2DResUnet. The DM-DA-Unet network based on the cascade mechanism requires distribution prediction. First, the entire image is predicted by 2DDenseUnet to obtain the three-dimensional boundary of glioma, the center of the box, and then use the center to take the 128*∗*128*∗*128 area as the input data of 3D DA-Unet, and finally use the 3D-DA-Unet area for predictive output, so as to obtain the final glioma output result.
6. The sixth step is the process of data postprocessing. On the basis of hole filling, the false positive core area that appears in the 3D-DA-Unet prediction result can be removed.

## 4. Experiment and Results Analysis

### 4.1. Data Set

In this article, in the process of experimental comparison of brain glioma segmentation algorithms, the BraTS17 data and BraTS18 data set in the BraTS data set are used as experimental data to train and verify related models. In the data set used in the experiment, the official training data of BraTS18 is divided into training set, test set, and validation set and used for local fivefold cross-validation. For the BraTS17 data set, the BraTS17 training set is used to train the two models proposed in this article, and the relevant models are evaluated online through the BraTS17 verification set.

### 4.2. Comparison with Other Methods

In order to better verify the effectiveness of the model, 2DUnet [25], 3DUnet [19], SegAN [26], Isensee 3DResUnet [27], and other models in related papers have been reproduced, and these models have been involved in experimental evaluation. Among them, 2DUnet is the original Unet structure using two-dimensional convolution. 3DUnet is the original Unet structure using three-dimensional convolution. The SegAN structure is a generative confrontation network that uses the Unet structure as a generator. Isensee 3DResUnet is a fully convolutional network with ResBlock mechanism added to 3DUnet. The experimental results are illustrated in Figures 5 and 6.

Through the evaluation results of the abovementioned fivefold cross-validation, it can be seen that the DM-DA-Unet model proposed in this paper has a significant improvement in various indicators compared with other models used in the experimental process.

Although the relevant models can be quantified and evaluated by locally dividing the data set and cross-validation, there is a problem that the amount of data is smaller than that of the real scene. Therefore, training overfitting may exist only through the verification method of locally dividing the data set. In order to alleviate this overfitting phenomenon and fully verify the robustness of the model, this article uses the BraTS2017 training set to train the 2DResUnet and DM-DA-Unet models proposed in this article. Then, the verification set of BraTS2017 was predicted, and the prediction results were submitted to the official website of BraTS2017 to obtain the results of online evaluation. Since the BraTS data set is widely studied, it can be compared and analyzed with the glioma segmentation model in related papers to objectively verify the effectiveness of the model. The related online evaluation results are shown in Table 1. Other methods include Zikic et al. [13], Pereira et al. [16], Havaei et al. [15], Naceur et al. [28], Wang et al. [29], Isensee et al. [27], and Kamnitsa et al. [30].

By comparing with the model evaluation results of other BraTS17 validation sets, the DM-DA-Unet structure proposed in this paper has significant segmentation effects on Dice Score, specificity, and sensitivity. The Dice Score of the best segmentation model on BraTS2017 has the same accuracy and is very close in other indicators.

Through the comparison results of the local cross-validation experiments and the evaluation results of the BraTS17 verification set submitted online, the following experimental analysis conclusions can be drawn.

In the evaluation results of the BraTS17 validation set, the glioma segmentation method using the full convolutional network is significantly better than the segmentation based on pixel-by-point segmentation on the three regions of glioma, including WT, CT, and ET. Convolutional network segmentation effect. And, in the BraTS data set, a fully convolutional network using three-dimensional convolution can achieve better segmentation effects than a fully convolutional network using two-dimensional convolution. By adding a feature extraction mechanism to the model, increasing the depth of the model, and using multiple models for integrated learning, the segmentation effect of the model can be effectively improved.

The DM-DA-Unet model proposed in this paper combines a two-dimensional fully convolutional network with a three-dimensional fully convolutional network through a cascade mechanism and uses the DenseBlock and Attention mechanisms. Thereby, the network structure and feature acquisition ability are improved, and the segmentation effect of glioma is significantly improved. In the local fivefold cross-validation process using the BraTS18 data set, the segmentation effect of this model is the best. Similar to the current best segmentation network in BraTS17, it can accurately segment gliomas in brain MRI.

## 5. Conclusion

The segmentation of glioma based on MRI can facilitate for doctors observation of the external morphology of each tumor tissue of the patient's glioma, and it is also helpful for doctors to analyze and treat the glioma based on imaging. This article mainly focuses on the research on the segmentation method of glioma based on deep learning and focuses on the description of the segmentation method of glioma based on full convolutional network. The main research contents and results are as follows: aiming at the problems that the current full convolutional network has two-dimensional convolution, it is difficult to obtain three-dimensional spatial information and the three-dimensional convolution consumes a lot of computing resources and so on; the DM-DA-Unet model is proposed. The model is a two-stage network with a cascading mechanism, and a full convolutional network of different dimensions is used in different stages. Different loss functions are used for training, and DenseBlock, Attention, and the mechanism of multiscale fusion in the upsampling process are used to improve the model. The proposed model was validated and evaluated. In order to objectively verify the effectiveness and robustness of the model, first use the BraTS18 data set for local fivefold cross-validation, then use the BraTS17 data set for online evaluation, and use four measurement methods to quantify the segmentation results of the model. The two proposed models and other glioma segmentation models currently proposed are compared and analyzed.

In the future, we are keen on extending the operational capacities of the proposed deep learning based method by combining it, specifically to form a hybrid model and use it for other purposes as well.

## Figures and Tables

**Figure 1:** DM-DA-Unet network structure.

**Figure 2:** Encoder DenseBlock structure.

**Figure 3:** Decoder DenseBlock structure.

**Figure 4:** Attention structure in DM-DA-Unet.

**Figure 5:** Dice Score and specificity of different methods.

**Figure 6:** Sensitivity and Hausdorff distance of different methods.

**Table 1:** Online evaluation results of the official verification set of Brats2017.

Method	Dice Score			Specificity			Sensitivity		
	WT	CT	ET	WT	CT	ET	WT	CT	ET
Zikic	0.84	0.74	0.69						
Pereira	0.87	0.73	0.68				0.86	0.77	0.70
Havaei	0.88	0.79	0.63				0.87	0.79	0.80
Naceur	0.89	0.76	0.81				0.82	0.82	0.69
Wang	0.88	0.82	0.74						
Isensee	0.89	0.79	0.73	0.99	0.99	0.99	0.89	0.82	0.80
Kamnitsa	0.90	0.79	0.73				0.90	0.78	0.76
Ours	0.90	0.80	0.73	0.99	0.99	0.99	0.89	0.77	0.75

## Data Availability

The data sets used and analyzed during the current study are available from the corresponding author upon reasonable request.
